RETRACTED

# Design, development, and evaluation of a registry system for hyperbaric oxygen therapy: A methodological study

**DOI:** 10.1002/hsr2.768

**Published:** 2022-08-08

**Authors:** Shahram Oliaei, Amirali Karimi, Ahmadreza Shamsabadi, Pegah Mirzapour, Hengameh Mojdeganlou, Zahra Nazeri, Amir B. Bagheri, Newsha Nazarian, Reyhaneh Jashaninejad, Mohammad Qodrati, Iman Amiri Fard, Farzaneh Ghanadinezhad, Arian Afzalian, Mohammad Heydari, Esmaeil Mehraeen, SeyedAhmad SeyedAlinaghi

**Affiliations:** ^1^ HBOT Research Center, Golestan Hospital, Islamic Republic of Iran Navy and AJA Medical University Tehran Iran; ^2^ School of Medicine Tehran University of Medical Sciences Tehran Iran; ^3^ Department of Health Information Technology Esfarayen Faculty of Medical Sciences Esfarayen Iran; ^4^ Iranian Research Center for HIV/AIDS, Iranian Institute for Reduction of High Risk Behaviors Tehran University of Medical Sciences Tehran Iran; ^5^ Department of pathology Urmia University of Medical Sciences Urmia Iran; ^6^ Department of Health Information Management Tehran University of Medical Sciences Tehran Iran; ^7^ Michael E. DeBakey Department of Surgery, Division of Vascular Surgery and Endovascular Therapy, Interdisciplinary Consortium on Advanced Motion Performance Baylor College of Medicine Houston Texas USA; ^8^ Faculty of Medicine Mashhad University of Medical Sciences Mashhad Iran; ^9^ School of Medicine Islamic Azad University Tehran Iran; ^10^ Department of Epidemiology, School of Public Health Hamadan University of Medical Sciences Hamadan Iran; ^11^ Iranian Research Center for HIV/AIDS, Iranian Institute for Reduction of High Risk Behaviors Tehran University of Medical Sciences Tehran Iran; ^12^ Department of Community Health Nursing and Geriatric Nursing, School of Nursing and Midwifery Iran University of Medical Sciences Tehran Iran; ^13^ Shahid Chamran University of Ahvaz Ahvaz Iran; ^14^ Department of Health Information Technology Khalkhal University of Medical Sciences Khalkhal Iran

**Keywords:** hyperbaric oxygen therapy, registry, registry systems, system development

## Abstract

**Background and Aims:**

Hyperbaric oxygen therapy (HBOT), utilizes 100% oxygen at pressures greater than sea‐level atmospheric pressure, for the treatment of conditions in which the tissues starve for oxygen. The Undersea and Hyperbaric Medical Society (UHMS) has granted HBOT approval for the treatment of various conditions. On the other hand, applying informatics registry systems can improve care delivery, ameliorate outcomes, and reduce the costs and medical errors for the patients receiving HBOT treatment. Therefore, we aimed to design, develop, and evaluate a registry system for patients undergoing HBOT.

RETRACTED

**Methods:**

In the first phase, the conceptual and logical models were designed after conducting symposiums with experts and having other experts review the models. In the second phase, the system was developed on the web using ASP.NET  and C# programming languages frameworks. The last phase involved Nielsen's heuristic evaluation method for the system's usability. Five experts evaluated the system, including three health information management specialists and two medical informatics specialists.

**Results:**

The hyperbaric patient information registry system (HPIRS) interacts with three types of users—a specialist physician, a nurse, and a system administrator. A scenario for each predefined activity was designed, and all the information was stored in the SQL servers. The five experts independently found 152 issues, of which 84 were duplicates. The 68 distinct issues of the system were then resolved.

**Conclusions:**

The design and development of such registry systems can make data available and stored carefully to improve clinical care and medical research and decrease costs and errors. These registries can provide the healthcare systems with E‐health applications, improved data management, more secure data transfer, and support for statistical reporting. The implemented heuristic evaluation method can also provide a low‐cost and readily available system to fix the issues of the designed systems.

## 1 INTRODUCTION

The first report on the therapeutic use of hyperbaric oxygen therapy (HBOT) was released in 1879 by the French surgeon Fontaine, who believed that pressurized oxygen chambers can help with anesthesia.^1^ Dr. Orville Cunningham also used HBOT and successfully treated a patient dying from the flu in 1918.^2^ Later on, in the 1950s and 1960s, Churchill‐Davidson and Boerma's work contributed to the recognition of the HBOT's effectiveness in the treatment of radiation therapy, anaerobic infections, carbon monoxide poisoning, and heart surgery.^3^ In terms of mechanism; HBOT therapy places the patients in a monoplace chamber, designed for only one patient, or a multiplace chamber, that can fit more than two patients, where they are exposed to 100% oxygen at higher than 1.4 atmosphere absolute (ATA) pressures to inhale. HBOT subsequently increases plasma and tissue oxygen levels significantly, which would be much lower at normal atmospheric pressures.^4^, ^5^ The duration of treatment varies based on the specific symptoms but is usually between 1.5 and 2 h.^6^, ^7^

HBOT can exert a variety of effects. It inhibits neutrophil adhesion and chemotaxis, halts proinflammatory cytokines production,^8^, ^9^ increases arterial O_2_ pressure,^10^, ^11^ alters the patient's microbiome metabolism, suppresses the formation of pro‐inflammatory mediators, decreases circulating lymphocytes and leukocytes,^12^ regulates the hypoxia response pathway, attenuates reperfusion injury, stimulates angiogenesis, assists with collagen matrix formation, promotes wound healing,^13^ and maintains allograft durability.^14^

RETRACTED

Based on all the biochemical effects mentioned above, HBOT has been proven to be safe and effective either alone or as an adjunct method in treating various diseases, with few side effects.^15^, ^16^ According to the Undersea and Hyperbaric Medicine Society (UHMS), HBOT is approved for the following indications; carbon monoxide poisoning, crushing traumas, compartment syndrome, cyanide intoxication, gas gangrene, decompression sickness, compromised skin graft, central retinal artery occlusion, osteomyelitis, delayed radiation injury, necrotizing soft tissue infection, air or gas embolism, actinomycosis, acute thermal burns, sensorineural hearing loss, anemia, and diabetic wounds.^15^ Possible adverse effects of HBOT are as follows: barotraumatic middle ear injury, sinus damage, oxygen poisoning‐which can cause pulmonary failure, pulmonary fluid congestion, seizures or myopia‐claustrophobia, hypoglycemia in diabetics, dizziness, and weakness.^17^, ^18^

Although, despite all the aforementioned therapeutic effects of HBOT, most of the available evidence regarding its efficiency is based on small‐scale randomized clinical trials (RCTs), and retrospective studies.^19^, ^20^ In addition, there is controversy in regard to its efficacy and actual place as a treatment of choice for in some studies.^21^ This controversy mostly stems from small‐sampled published articles and the difficulties researchers face conducting large‐sampled trials. Also, although many national‐scale policy‐making agencies like US Food and Drug Administration (FDA) have granted safety and efficacy approval to hyperbaric oxygen chambers for a wide range of conditions,^22^ others like National Health Service (NHS) have only granted HBOT approval for decompression illness and gas embolism treatment.^23^ Additionally, HBOT study and research have its own particular difficulties because; it is a long‐standing treatment process with a daily session for a few months, and most centers do not have enough numbers of engaged cases to form a reasonable sample size and carry out a research study, and most patients are followed by other specialties so their outcomes are mostly unavailable.^6^ Thus, to gather information regarding HBOT outcomes, long‐term follow‐up, and efficacy assessment a multicenter computerized data collection system is needed. One high‐yield system is the registration system that is used in hospitals and clinics to record information about patients with specific conditions. The registry is the systematic data collection on specific diseases, such as cancer, and AIDS.^24^, ^25^, ^26^ The database of this system contains uniform information about patients, collected systematically and comprehensively for scientific research and clinical services with a predefined policy.^27^, ^28^ This system is an ideal tool for clinical study when outcome assessment and treatment guideline policy making is essential. In many diseases, recording systems are used for epidemiological, preliminary, and risk modeling studies.^29^ Therefore, we aimed to design, develop, and evaluate a registry system for patients undergoing HBOT to address the gaps in regard to its safety, efficacy, and outcomes.

RETRACTED

## 2 METHODS

This methodological study has three phases. Tehran University of Medical Sciences and Golestan hospital were the sites of the study. In the first phase: Conceptual and logical models of different parts of the information system of hyperbaric patients were developed by using the results of the first phase of the research and holding symposiums with specialists (8 physicians, 15 nurses, and 1 health information management). Objectives, mainstream events, preconditions processes, and background conditions were discussed in these symposiums. Then the system's conceptual model was designed in the form of Unified Modeling Language (UML) diagrams, including class diagrams, use case diagrams, and activity diagrams using Microsoft Visual software. Finally, the conceptual and logical models of the system were reviewed by experts, the corrective comments and suggestions were received, and the desired changes were applied.

In the second phase: We developed and implemented the development system of the Hyperbar Patient Information Registration System on the web using the ASP.NET Framework and in the C# programming language in the NET Framework 4.5 technology platform. The SQL Server database was also used to store information.

In the third phase: The Nielsen evaluation method evaluated the system's usability. This evaluation includes 10 principles for examining user interface design problems and is performed by trained professionals to identify and eliminate defects and create effective interaction between the user and the system. This method evaluates a system based on design principles, including system status visibility, user control, compatibility, standards, flexibility, and efficiency.^30^ In this study phase, three health information management specialists and two trained medical informatics specialists familiar with Nielsen's 10 evaluation principles were selected to independently examine the assessment of different parts of the hyperbaric patient information registration system in terms of 10 principles Nielsen. After identifying the problems by each evaluator, duplicate cases were eliminated, and similar cases were identified. To evaluate the usability of the system, the Nielsen 10 Principles Checklist was used, which is usually used for exploratory evaluation. After evaluating the system by experts, problems were identified by each of them. The severity of the problem was then ranked from zero to four based on the Nielsen checklist. Finally, repetitive cases were eliminated and similar cases were identified. Data analysis was performed with SPSS version 21. Results are consulted with statistics and IT specialists (Table 1).

RETRACTED

**Table 1:** Problem rating scale based on Nielsen exploratory evaluation model^6^

Score = 0 and average intensity = 0–0.5	Without problem–no problem
Score = 1 and average intensity = 0.6–1.5	Minor problem–no need to correct the problem
Score = 2 and average intensity = 1.6–2.5	Small problem–low priority problem correction
Score = 3 and average intensity = 2.6–3.5	Big problem–high priority problem correction
Score = 4 and average intensity = 3.6–4	Serious problem–high need for problem correction

## 3 RESULTS

### 3.1 Designing phase

The UML diagrams and Microsoft Visio were used to model the hyperbaric patient information registry system (HPIRS). The HPIRS interacts with three types of users—the specialist physician, the nurse, and the system administrator, and provides each of them with some features based on their defined roles and access levels (Table 2 and Figure 1).

**Table 2:** Identifying roles of HPIRS users

No.	User	Roles
1	Specialist physician	Register into the system Log‐in to the system Record clinical data Demonstrate recorded data and debrief on treatment plan Present medication and laboratory orders Log‐out of the system
2	Nurse	Register into the system Log‐in to the system Record admission and clinical data Demonstrate of recorded data and debrief on treatment plan Log‐out of the system
3	System administrator	Register into the system Log‐in to the system Control of user access level Edit user profiles Generate reports from the system Log‐out of the system

Abbreviation: HPIRS, hyperbaric patient information registry system.

**Figure 1:** Use case diagram for the hyperbaric patient information registry system user

To determine the activities of the HPIRS, a scenario related to each activity was presented. Table 3 shows the scenario related to user registration in the HPIRS.

RETRACTED

**Table 3:** The scenario for registration in the HPIRS

Use case name	Register	
Scenario	Registration of the user into the system.	
Brief description	Through this use case, the user enters and submits their identity information as well as a username and password.	
Actors	Specialist physician, nurse, and system administrator.	
Preconditions	Users must have been accepted by the system administrator before they were able to login to the system.	
Postconditions	The user's identity information, username, and password are saved. S/he is registered into the system.	
Workflow	Actor	System
	− User runs the application. − User requests the registration form. − User enters identity information, username, and password. − User presses the “submit” button.	− The system displays the identity information form. − The system checks the entered information. − The system saves the user identity information. − The message “successfully registered” is shown.
Exceptions	− If the user clicks the “back” button in any step, the system will exit without any changes. − If the system encounters a problem saving the information, it will display the message and will exit the form without any changes.	

Abbreviation: HPIRS, hyperbaric patient information registry system.

### 3.2 Developing phase

Microsoft Windows was used to develop the HPIRS, and SQL Server was preferred to provide databases for data persistence. The architecture of the HPIRS is shown in Figure 2.

**Figure 2:** Architecture of the HPIRS

To develop HPIRS, first, the programming language and its appropriate database were investigated. Because the system was web‐based, the ASP.NET programming language was used. SQL Server was used to develop the database in Visual Studio infrastructure. The HPIRS is web‐based and does not require software installation and so users can access the system through all browsers after specifying the username and confirming access.

### 3.3 Evaluation phase

The HPIRS was evaluated by Nielsen's heuristic evaluation. In this method, evaluators (three health information management specialists and two medical informatics specialists) evaluated the system. The evaluators identified 152 issues in different areas. Each of the evaluators independently found 29 (19.07%), 29 (19.07%), 30 (19.73%), 31 (20.39%), and 33 (21.71%) issues. After the exclusion of 84 duplicates, 68 individual issues were investigated and then resolved.

As shown in Table 4, among the identified issues, the most common ones were related to the item of “help and documentation” (19.11%) and “consistency and standards” (13.23%). The least problems were related to the item of “flexibility and efficiency of use” (4.41%) and “esthetic aspects and simple design” (4.41%).

RETRACTED

**Table 4:** Identified issues according to the 10 principles of Nielsen heuristic evaluation

No.	Items	Totla number of identified problems (%)	Mean of severity ratings	Number of identified problems					Severity
				E. 1	E. 2	E. 3	E. 4	E. 5	
1	Visibility of system status	7 (10.29)	0.4	2	2	2	0	1	Without problem
2	Match between system and the real world	6 (8.82)	0.5	1	1	0	2	2	Without problem
3	User control and flexibility	8 (11.76)	0.2	2	3	2	1	0	Without problem
4	Consistency and standards	9 (13.23)	1.31	3	2	1	2	1	Partial problem
5	Help to errors recognize and correction	8 (11.76)	2	4	0	1	1	2	Minor problem
6	Error prevention	5 (7.35)	1.74	1	1	0	0	3	Minor problem
7	Recognition rather than recall	6 (8.82)	1.56	1	2	1	1	1	Partial problem
8	Flexibility and efficiency of use	3 (4.41)	0.4	2	1	0	0	0	Without problem
9	Esthetic aspects and simple design	3 (4.41)	0.3	0	0	1	1	1	Without problem
10	Help and documentation	13 (19.11)	2.9	3	3	4	2	1	Major problem
Total		68 (100)	1.13	19	15	12	10	12	Partial problem

Abbreviation: E, evaluator.

## 4 DISCUSSION

Investing in information technology in the field of health today has opened up new avenues for healthcare evolution. As a result, developing a patient information registration system could be extremely valuable to both healthcare providers and patients both during and after treatment. Soft tissue injuries, wound healing, and underwater medicine are only a few of the indications for HBOT.^6^, ^31^ recent research has revealed that hyperbaric oxygen treatment is effective in the treatment of a number of ailments. The development of a patient information registration system for undersea medicine and HBOT could be advantageous.^32^

The primary purpose of information registration systems in healthcare centers is to record and compare patients’ information and to be able to check and compare the condition of patients before and after using a treatment method. Creating the minimum set of data elements is one of the essential steps in developing any information system; It allows data from many organizations, institutions, and information systems to be matched to ease data comparison and determine the information needs of users.^32^ Accuracy and completeness of data are the most critical factors affecting the quality and value of any registration system.^6^, ^16^, ^31^, ^32^

This system has three types of actors: a specialist physician, a nurse, and a system administrator, each with their own set of responsibilities. Data from various locations can be recorded at the same time using this user‐friendly web‐based registry system. It is both cheap and time intensive. It also makes it simple to update data and share it.^6^

RETRACTED

Some studies evaluate a web‐based system designed in a Visual Studio environment with C# program language with NET 4.5 technology framework. The database was designed in SQL server 2016. Some other studies also used the mentioned software and programming language for creating and implementing their web‐based system, which provided the necessary connection and integration between the server, programming, data access, and security tools.^25^, ^33^, ^34^

The results of other studies from Iran indicated that web‐based logging systems increase the accuracy and speed of data entry and reduce the risk of errors along with lower cost; in addition, web‐based registration systems facilitate updating information, creating complex reports, and sharing information.^35^, ^36^

An essential part of any system management is evaluation, which examines the performance of the system to assess the achievement of goals. Through the results obtained from the evaluation of information systems, it is possible to identify the strengths and weaknesses of the systems, which increase the quality of care services and improve the appropriate decision‐making. Existing problems are identified through the evaluation of information systems and based on the findings, necessary corrective actions are taken. The most crucial point in evaluating health systems is to perform the evaluation process with sufficient speed and accuracy, and finally, to solve problems.^37^

The HPIRS was evaluated by Nielsen's heuristic evaluation. The evaluators identified 152 issues in different areas. After excluding 84 duplicates, 68 identical issues were investigated and then resolved. Among the identified issues, the most common ones were related to the item of “help and documentation” (19.11%) and “consistency and standards” (13.23%). Minor problems were related to the item of “flexibility and efficiency of use” (4.41%) and “esthetic aspects and simple design” (4.41%). Considering the different goals of information systems for applied research, nonrepetition of activities and reduction of costs, management of health systems, and increasing the quality of care and health services, continuous evaluation of these systems is important.^38^ A similar study showed that the most usability problems of health information systems were related to heuristics of help and documentation.^39^

Hadanny et al. evaluated the safety of hyperbaric oxygen treatment and found out that 17.4% of patients treated with hyperbaric oxygen experienced an adverse event. And the most complication was barotraumas to the ear. They concluded that with some evaluations before and after therapy and also patient monitoring that the patients' safety improves. This shows the necessity of a registry system that helps us to register patients’ evaluation data and monitoring.^40^

RETRACTED

A consistent study by Harlan et al. showed that by establishing a registry system, information from multiple centers can be collected. By expanding this system, more detailed data could be gathered and long‐term follow‐up is feasible.^6^ The systematic review of Poffley et al. evaluated the national and international registries on cardiac rehabilitation. They showed that the use of registries for cardiac rehabilitation provides quality improvement, especially in the early stage.^32^

Our study also focused on reviewing the design of the registry system, evaluating the development of the model and its different phases, and assessing the costs, issues, and problems of this system. Different programming languages, networks, and databases were implemented to evaluate and appraise the different aspects of this model. The present study has some benefits; its novelty is a critical strength and similar studies with a focus on HBOT are few. Also, evaluating and recognizing the most important problems of the hyperbaric registry systems is one of the essential study goals which is one of the practical aspects of our study.

But the study has some limitations; as this registry system is almost new, the data about this system is limited. As mentioned before, a checklist was used for the problems. But there may be some problems out of the checklist, this is another limitation of our study. Also, we could not evaluate the system's effectiveness; this section needs more studies in the future. We also evaluated this system for a particular treatment, although the registry systems can be used for other diseases and treatments. Putting all together, by maintaining a complete and reliable data record, and further evaluation, this clinical data registry reduces bias. With this technique, practitioners have access to a large amount of accurate data through a web‐based system, in an organized style, allowing them to compare the treatment process and outcome of therapy with other practitioners to enhance their work and reach optimal performance.^41^

Because hyperbaric oxygen treatment requires numerous sessions, which might take several months, this registry system allows practitioners to record multiple data in an organized manner, and the pooled data assists practitioners in evaluating therapy outcomes and patient prognosis. Patients may be better tracked throughout their treatment with this technique, and it also allows for more robust research ^6^ E‐health applications, improved data management, more secure data transfer, and support for statistical reporting. Registration systems are becoming more widely recognized as useful, accurate, and dependable methods for assessing the diversity of service and improving quality in healthcare systems. This system allows specialists to more correctly identify clinical and laboratory symptoms, respond to treatments, outcomes, and problems, and improve diagnostic and therapeutic decisions for patients.^6^, ^41^

RETRACTED

## 5 CONCLUSION

The article explains the data elements and technical requirements of the HBOT patient information registration system. Also, it includes the steps in designing in addition to creating a patient information registry in the same subject. It clarifies the evaluation of the results of the hyperbaric patient information registration system. During this research a lot of important complications have been recognized, which was one of its main targets.

At last, a vivid point of this article that values the study is the novelty of the subject and there are a few other research studies in this field. In conclusion, considering the expansion of information technology goals and their increasing application in the field of information management, it is suggested for future studies to expand and develop a registry system through which, the healthcare provider could have online access all over the world. More studies are also recommended to identify the requirements for designing and developing an information registration system for other clinical areas including cardiovascular, renal diseases, and cancers. Also, to evaluate the cost and benefit of using a hyperbaric therapy registration system, and assess the benefits of using hyperbaric therapy information registration system on the quality of patient care, and the rate of morbidity and mortality and finally to do more research and evaluation on long‐term follow up of the patients using this system.

## AUTHOR CONTRIBUTIONS

**Shahram Oliaei**: Conceptualization. **Amirali Karimi**: Formal analysis. **Ahmadreza Shamsabadi**: Formal analysis. **Pegah Mirzapour**: Formal analysis. **Hengameh Mojdeganlou**: Formal analysis. **Zahra Nazeri**: Writing—original draft; writing—review and editing. **AmirBehzad Bagheri**: Writing—original draft; writing—review and editing. **Newsha Nazarian**: Writing—original draft; writing—review and editing. **Reyhaneh Jashaninejad**: Writing—original draft; writing—review and editing. **Mohammad Qodrati**: Writing—original draft; Writing— review and editing. **Iman Amiri Fard**: Writing—original draft; writing—review and editing. **Farzaneh Ghanadinezhad**: Writing—original draft; Writing—review and editing. **Arian Afzalian**: Writing—original draft. **Mohammad Heydari**: Methodology; writing—original draft. **Esmaeil Mehraeen**: Conceptualization; writing—original draft. **SeyedAhmad SeyedAlinaghi**: Conceptualization; writing—original draft.

RETRACTED

## CONFLICT OF INTEREST

The authors declare no conflict of interest.

## TRANSPARENCY STATEMENT

The lead author (Esmaeil Mehraeen) affirms that this manuscript is an honest, accurate, and transparent account of the study being reported; that no important aspects of the study have been omitted; and that any discrepancies from the study as planned (and, if relevant, registered) have been explained.

## ETHICS STATEMENT

The current study was extracted from the study project with code RLT‐B 1514 entitled “Design, Development and assessment of Comprehensive Registry System for Submarine, Diving and Hyperbaric Medicine” conducted at Supreme National Defense University in 2021.

## Data Availability

The authors confirm that the data supporting the findings of this study are available within the article [and/or] its Supporting Information.
